The article "Synthesis and Evaluation of Finasteride-Loaded HPMC-Based Nanogels for Transdermal Delivery: A Versatile Nanoscopic Platform" was retracted in 2024. Reasons: signs of a paper mill; compromised peer review; unreliable results or conclusions.

# Synthesis and Evaluation of Finasteride-Loaded HPMC-Based Nanogels for Transdermal Delivery: A Versatile Nanoscopic Platform

**DOI:** 10.1155/2022/2426960

**Published:** 2022-07-19

**Authors:** Aousaf Ahmad, Mahmood Ahmad, Muhammad Usman Minhas, Muhammad Sarfraz, Muhammad Sohail, Kifayat Ullah Khan, Sana Tanveer, Shakeel Ijaz

**Affiliations:** ^1^Department of Pharmaceutics, Faculty of Pharmacy, The Islamia University of Bahawalpur, 63100 Punjab, Pakistan; ^2^Quaid-e-Azam College of Pharmacy, Sahiwal, Punjab, Pakistan; ^3^College of Pharmacy, University of Sargodha, University Road Sargodha City, Punjab, Pakistan; ^4^College of Pharmacy Al Ain University, Al Ain Campus, Al Ain, UAE; ^5^Department of Pharmacy, COMSATS Institute of Information Technology, Abbottabad, 22060 KPK, Pakistan

## Abstract

Herein, we report nanogels comprising diverse feed ratio of polymer hydroxypropyl methylcellulose (HPMC), monomer acrylic acid (AA), and cross-linker methylene bisacrylamide (MBA) fabricated for transdermal delivery of finasteride (FIN). Free radical solution polymerization method with subsequent condensation was employed for the synthesis using ammonium per sulfate (APS) and sodium hydrogen sulfite (SHS) as initiators. Carbopol-940 gel (CG) was formulated as assisting platform to deliver FIN nanogels transdermally. Developed formulations were evaluated by several *in vitro*, *ex vivo*, and *in vivo* parameters such as particle size and charge distribution analysis, Fourier transform infrared spectroscopy (FTIR), thermogravimetric analysis (TGA), differential scanning calorimetry (DSC), scanning electron microscopy (SEM), X-ray diffractogram (XRD), rheological testing, *in vitro* swelling and drug release, and *ex vivo* skin permeation, irritation, and toxicity assessment. The results endorsed the nanogel formation (117.3 ± 29.113 nm), and the impact of synthesizing method was signified by high yield of nanogels (≈91%). Efficient response for *in vitro* swelling and FIN release was revealed at pH 5.5 and 7.4. Skin irritation and toxicity assessment ensured the biocompatibility of prepared nanocomposites. On the basis of the results obtained, it can be concluded that the developed nanogels were stable with excellent drug permeation profile across skin.

## 1. Introduction

Nanogels are basically hydrogels of nanoregime, usually composed of polymeric backbone-based cross-linked network [1, 2]. Bearing the features of hydrogels with added scope of nanoscale particle size, they overcome drawbacks of micro- and macroscale hydrogels [3]. Tuning and optimization of molecular composition, size, and design of nanogels can yield several advantages, i.e., stimuli responsive, easy and efficient drug loading, remarkable permeation across biological barriers, improved drug release profile, biocompatibility, and physical stability of the system [4, 5]. Due to their wide range of properties, nanogels can encapsulate diverse classes of bioactive materials. Nanogels of polyelectrolyte origin can swiftly capture opposite charged low molecular weight drugs. Drug molecules develop electrostatic interaction and bound in charged network of the system. Mentioned properties help in the formation of a product for biomedical application that aids in improving patient compliance [6, 7].

The article "Synthesis and Evaluation of Finasteride-Loaded HPMC-Based Nanogels for Transdermal Delivery: A Versatile Nanoscopic Platform" was retracted in 2024. Reasons: signs of a paper mill; compromised peer review; unreliable results or conclusions.

Benign prostatic hyperplasia (BPH) is a common, progressive androgen-dependent disease in aging men resulting in an enlargement of prostate which in turn can lead to obstruction of urethral lumen and even complete urinary retention [8, 9]. Finasteride (FIN) is a selective 5-*α*-reductase inhibitor, reduces the conversion rate of testosterone to dihydrotestosterone which is a major cause of BPH, thus reducing the prostate size and improving the urinary symptoms. Persistent reduction in prostate size by FIN therapy can prevent BPH progression and prostate cancer as well [10, 11]. In effective treatment plan of BPH, FIN is continuously prescribed for months by oral route. FIN is also reported for its low oral absorption and bioavailability [12]. As BPH is associated to old age group majorly, long-term therapy of FIN potentially with other drugs also can produce gastric discomfort [13, 14].

Drug delivery by transdermal route provides an alternative way to avoid such complications. By TDDS, higher drug permeation can be achieved due to prolonged contact onto or within layers of skin channels [15]. Hydrogel nanoparticles of biocompatible profile and being of nanoscale can be highly effective in achieving effective treatment by transdermal route [16, 17]. Physicochemical characteristics along with pharmacokinetic and pharmacodynamics profile of drugs are taken as top list factors in designing of drug delivery systems. With emerging novelty and developing efficacious therapy measures, several limitations of conventional systems, i.e., poor pharmacokinetics and toxicity, can be reduced [18]. Ideal candidates for TDDS are characterized by lower molecular weight, optimum lipophilicity, and higher potency. Meeting the said criterion, transdermal route is favorable for molecules having short t_1/2_, poor oral absorption, and bioavailability [19].

HPMC is a white, odorless surfactant of nonionic origin. Nanogels are composed of ionic/nonionic network of amphiphilic polymer chains, when dispersed in aqueous media swell to considerable volume and can load efficient amount of drug. Due to its properties, it possesses promising window to be used in biocompatible drug carrier systems [20, 21]. Acrylic acid is a monomer of liquid origin. Due to its physicochemical profile and reactivity, it has tremendous potential to be used in nanogel synthesis. In literature, it has been reported as a constructive part of nanogel design [22, 23].

The article "Synthesis and Evaluation of Finasteride-Loaded HPMC-Based Nanogels for Transdermal Delivery: A Versatile Nanoscopic Platform" was retracted in 2024. Reasons: signs of a paper mill; compromised peer review; unreliable results or conclusions.

In the context of the above information, the present study was focused to prepare and characterize HPMC-based nanogels loaded with FIN as a model drug in order to overcome the issues of poor absorption and bioavailability as well as to improve the patient compliance regarding long-term therapy. Manuscript being a bridge of hydrogels and nanoclass systems was aimed at summarizing the output of various *in vitro*, *ex vivo*, and *in vivo* parameters emphasizing nanogels for safe and efficacious transdermal delivery.

## 2. Materials and Methods

### 2.1. Materials

Finasteride was received as kind gift from Linear Pharma, Pakistan. HPMC 15 Cps and acrylic acid were obtained from Sigma-Aldrich, USA. Ammonium per sulfate (APS), sodium hydrogen sulfite (SHS), sodium hydroxide (NaOH), potassium dihydrogen phosphate (KH_2_PO_4_), and methylene bisacrylamide (MBA) were procured by Merck KGaA, Germany. Analytical grade solvents were utilized for the experimental work.

### 2.2. Methods

#### 2.2.1. Formulation of HPMC-Co-AA Nanogels

A modified aqueous based free radical polymerization method was adopted for the fabrication of HPMC-co-acrylic acid nanogels [24]. To make HPMC solution, 2/3 of the required distilled water was kept at hot plate magnetic stirrer with temperature maintained at 70°C. The required amount of polymer was added slowly into hot water with continuous stirring at 250 rpm. Temperature was dropped gradually, and the remaining distilled water was added slowly which resulted in the formation of a thick solution. Meanwhile, aqueous solution of APS/SHS was added in AA at 250 rpm, and this mixture was then poured slowly to polymer solution at 700 rpm. Resultant mixture was homogenized by high speed homogenizer for 15 minutes at 11000 rpm with subsequent sonication and purging of nitrogen gas to remove dissolved air. MBA was dissolved in distilled water separately at 50°C. This was added dropwise to the above mixture at 1000 rpm and instantly channelized for gelation to already setup condenser maintained at 85°C. The whole mixture was allowed to condense for 4-5 h. The obtained formulation was subjected for approximately five minutes to the ethanol-water mixture (50 : 50) to get rid of unreacted constituents. Finally, formulation was sieved and kept in oven for 35–40°C for 48 h to get dried. Various ratios of polymer, monomer, and cross-linker were employed for fabrication of HPMC-based nanogels as shown in Table 1.  Figure 1 explains the possible nanogel network structure.

The article "Synthesis and Evaluation of Finasteride-Loaded HPMC-Based Nanogels for Transdermal Delivery: A Versatile Nanoscopic Platform" was retracted in 2024. Reasons: signs of a paper mill; compromised peer review; unreliable results or conclusions.

#### 2.2.2. Drug Loading

Drug loading in nanogel composites was carried by adapting swelling-diffusion method [25]. 2% (*w*/*v*) FIN solution was prepared in a mixture of ethanol-water (50 : 50). The purpose to use mixture of ethanol and water was to rationalize the solubility of the drug and to promote the swelling of nanogels. Accurately weighed dried nanogels were immersed in calculated volume of drug solution and allowed to stand for 24 h at room temperature. Drug-loaded nanogels were first dried at room temperature and then subjected to lyophilization for freeze drying.

#### 2.2.3. Preparation of Carbopol-940 Gel

For the preparation of a gel as a platform to spread hydrogel nanoparticles on skin, 0.6% carbopol-940 solution was prepared by dispersing calculated mass of gelling agent in distilled water at magnetic stirrer for 15-20 minutes while maintaining the rotation speed at 300 rpm. The gel was then made viscous and pH adjusted to 5.5 by using few drops of triethanolamine (TEA).

#### 2.2.4. Percent Yield

The efficiency of method was evaluated by calculating percentage yield of all formulations. Percent yield was measured by the following formula:

(1) $$\begin{array}{c} \text{Percent yield}=\frac{\text{Practical yield }}{\text{Theoretical yield}}\times 100. \end{array}$$

#### 2.2.5. FTIR Spectroscopy

FTIR spectroscopy using Bruker FTIR (Tensor 27 series) was employed for structural analysis and drug-formulation interaction by applying attenuated total reflectance (ATR) technology [26, 27]. Spectra of optimized loaded, unloaded formulation, and their pure components were obtained between scanning range of 400 and 4000 cm^−1^, and the recorded data was processed by OPUS Software (Bruker).

#### 2.2.6. Particle Size and Zeta Potential Analysis

Particle size and charged distribution of optimized formulation were determined using laser light scattering particle size analyzer (Malvern Zetasizer Nano ZS, UK). 0.1% (*w*/*v*) of nanogel dispersion was made with acetone. Homogenous suspension obtained was examined for particle size and zeta potential.

#### 2.2.7. Thermal Analysis

Thermal stability was studied by thermogravimetric analysis and differential scanning calorimetry using TA (Q600 Series, USA). Thermogravimetric analyzer was used to determine the rate and extent of weight change relative to temperature. Initially, reference standards were used to calibrate the weight profile. A known weight (0.5 to 5 mg) of the HPMC, FIN, and prepared formulation was placed in crimped aluminum pans in crucible baskets. The samples were analyzed at a scanning rate of 10°C/min from 0°C to 500°C under inert nitrogen flow rate of 10 ml/min to measure percent weight loss with increasing temperature. Differential scanning calorimetry (DSC) of HPMC, FIN, and developed formulation was used to evaluate melting point with respect to free energy absorbed and released. Sapphire standard was used for the calibration of calorimeter for heat capacity. Indium was used as a standard for cell constant and temperature [28].

The article "Synthesis and Evaluation of Finasteride-Loaded HPMC-Based Nanogels for Transdermal Delivery: A Versatile Nanoscopic Platform" was retracted in 2024. Reasons: signs of a paper mill; compromised peer review; unreliable results or conclusions.

#### 2.2.8. X-Ray Diffraction Analysis

Optimized formulation along with its constituents was subjected to XRD analysis using X-ray diffractometer (JDX3522, Japan). Tightly packed samples in aluminum cells were exposed to CuKa radiations of wavelength 1.54056 A°. Powder X-ray diffractograms were taken at 2Ɵ value up to 60. Operating conditions were 1 sec (count time), 0.050° (step angle), 2.5–30 mA (tube current), and 20-40 kV (tube voltage). The X-ray patterns recorded were then analyzed to study the crystalline/amorphous nature of samples [29, 30].

#### 2.2.9. Scanning Electron Microscopy

The surface morphology and shape of nanogels were examined using scanning electron microscopy (JSM5910, Japan). Optimized sample was prepared by sprinkling the formulation on a double-adhesive tape stuck to an aluminum stub. The stub was then coated with gold using a gold sputter module in a high-vacuum evaporator to a thickness of ~300 Å under an argon atmosphere.

#### 2.2.10. In Vitro Swelling Studies

Nanogel particles of known weight were placed in dialysis membrane and then immersed in phosphate buffer maintained at pH 5.5 and 7.4. They were allowed to swell; membranes from buffer were removed and weighed again after blotting. The difference in weight was calculated in order to observe the swelling of nanogels. The swelling ratio (SR) was calculated using the following formula [31]:

(2) $$\begin{array}{c} \text{Swelling Ratio}=\frac{W_{s}}{W_{d}}, \end{array}$$

where *W*_*s*_ represents the weight of swollen state of sample and *W*_*d*_ is the weight of sample in the dry state.

#### 2.2.11. Drug Entrapment Efficiency

The percent drug entrapment efficiency (DEE %) of developed nanogels was calculated by absorption and extraction method. Nanogels were weighed (100 mg) with accuracy and mixed in 50 ml of acetonitrile. This mixture was kept at magnetic stirrer with rotation speed of 100 rpm for 1 hour at room temperature. Obtained suspension was filtered using 0.45 *μ*m membrane filter. Filtrate was checked by UV spectrophotometric analysis at *λ* max 210 nm, and following formula was applied for quantitative estimation of entrapment efficiency.

(3) $$\begin{array}{c} \%\text{Drug Entrapment Efficiency}=\frac{\text{Actual Drug in Formulation }}{\text{Theoretical Drug in Formulation}}\times 100. \end{array}$$

The article "Synthesis and Evaluation of Finasteride-Loaded HPMC-Based Nanogels for Transdermal Delivery: A Versatile Nanoscopic Platform" was retracted in 2024. Reasons: signs of a paper mill; compromised peer review; unreliable results or conclusions.

#### 2.2.12. In Vitro Drug Release Studies

*In vitro* release studies of FIN from all loaded formulations were evaluated using USP Apparatus-V (paddle over disc method) with tea bag method [32]. Accurately weighed formulations were enclosed in emptied tea bags, and discs were placed in dissolution medium. The medium was composed of buffer maintained at pH 5.5 and 7.4 to simulate with pH of the skin and blood, respectively. For pH 5.5, apparatus was maintained at 32°C ± 0.5°C, while for 7.4 pH, it was maintained at 37°C ± 0.5°C with rotation speed of 50 rpm. Samples were withdrawn up to 120 minutes at specific internals of 10, 20, 30, 60, 90, and 120 minutes using a pipette and further diluted, and the amount of drug release was analyzed using UV spectrophotometer at *ʎ* max 210 nm.

#### 2.2.13. Sol-Gel Fraction Analysis

Nanogels were analyzed for sol and gel fraction using Soxhlet extraction setup where nanogels were kept for 4 hours with water at 80°C. Recollected nanogels were dried in vacuum oven at 45°C till constant mass. The following formulas were applied to calculate the sol and gel fractions.

(4) $$\begin{array}{c} \%\text{Sol Fraction}=\frac{W_{0}-\text{wt}}{W_{0}}\times 100, \end{array}$$

(5) $$\begin{array}{c} \%\text{Gel Fraction}=100–\text{Sol Fraction}, \end{array}$$

where in sol fraction, *W*_0_ is weight of nanogels before extraction and wt is weight after extraction.

#### 2.2.14. Porosity Analysis

Percent porosity (%) of nanogels was measured by fluid displacement method. Initially, preweighed oven dried nanogels were immersed in distilled water till saturation, and change in weight was marked. Saturated nanogels were blotted and weight variation was calculated. The following mathematical tool was employed to calculate % porosity.

(6) $$\begin{array}{c} \%\text{Porosity}=\frac{\text{Ws}-\text{Wd }}{\rho V}\times 100, \end{array}$$

where Ws is the weight of saturated nanogels, Wd is the weight of dried nanogels, *ρ* is the distilled water density, and *V* is the volume of respective formulation.

#### 2.2.15. Rheology and Stability of Gel

Programmable rheometer (Brookfield DV-III ultra) was used to study the viscoelastic behavior of the gel. Data analysis was carried out with Rheocalc V.2.010. Prior to each reading, gel samples were equilibrated. Continuous shear investigation was done with rheometer having CP41 spindle with cone and plate geometry as a measuring system. Shear rate was increased in ascending order as well as in descending order from 0 to 60 D in order to obtain up and down curves. The resultant shear stress was measured accordingly. In order to access the stability of gel formulation, samples were stored at the temperature of 8, 25, 32, and 45°C for three months.

The article "Synthesis and Evaluation of Finasteride-Loaded HPMC-Based Nanogels for Transdermal Delivery: A Versatile Nanoscopic Platform" was retracted in 2024. Reasons: signs of a paper mill; compromised peer review; unreliable results or conclusions.

#### 2.2.16. Ex Vivo Skin Permeation Studies

*Ex vivo* permeation studies were carried out using excised skin of rabbit. Animals were sacrificed employing an anesthetic agent. Abdominal hair along with fat adhered to dermis was removed by using hair removing cream. Finally, the skin was rinsed with phosphate buffer (pH 7.4). Prepared skin samples were stored in a refrigerator at –20°C and used within 24 hours. FIN *ex vivo* permeation through excised rabbit skin was performed using Franz diffusion cell consisting of two compartments, donor and receptor. The excised skin was mounted between both compartments. Phosphate buffer (pH 7.4) was used as receptor medium. The entire setup was placed over magnetic stirrer, with temperature maintained at 37 ± 0.5°C. After the hydration of excised skin, nanogels were applied on it. A specified volume of medium was collected and replaced with fresh medium. Amount of permeated gel was analyzed using UV spectrophotometer. The sample was collected up to 24 hours at specific intervals of 2, 4, 6, 8, 12, 18, and 24 hours, and then, the amount of drug in permeated samples was calculated. All surgical and experimental procedures had been reviewed and approved by the institute's Pharmacy Research Ethics Committee (PREC).

#### 2.2.17. Skin Irritation and Toxicity Studies

Skin irritation and toxicological studies were conducted on albino rabbits for assessment of dermal irritation and toxicological effects. All the procedures were conducted according to the Economic Co-operation and Development (OECD) guidelines and by the approval of institute's Pharmacy Research Ethics Committee (PREC). Rabbits weighing 2–2.5 kg were taken randomly and divided into two groups, i.e., G-1 and G-2, with three rabbits each (*n* = 3). The test animals were caged individually. 24 hours prior to the experiment, dorsal surface of rabbits was shaved properly with depilatory cream. Hair-free surface was marked with an area of approximately 5 cm^2^. The rabbits were treated as follows:

Test formulation of about 500 mg/kg was applied to the respective area. Observations were made after a period of 24, 48, 72, and 240 hours. On regular basis, animals were physically examined to observe and note any variance in skin appearance, body weight, eating pattern, amount of water and food consumption, sleep habits, salivation, diarrhea, and mortality. Blood of the rabbits was taken for biochemical analysis. Organs, i.e., the kidney, heart, lungs, liver, and spleen, were removed, weighed, and kept in suitable containers with formalin. Slides for histological examination were made. Optical microscope (Nikon E200, japan) with camera and software (MINISEE) was used to record histopathological images from slides.

The article "Synthesis and Evaluation of Finasteride-Loaded HPMC-Based Nanogels for Transdermal Delivery: A Versatile Nanoscopic Platform" was retracted in 2024. Reasons: signs of a paper mill; compromised peer review; unreliable results or conclusions.

Group 1: control group (blank without any test formulation)

Group 2: CG with HPMC-based nanogels

## 3. Result and Discussion

### 3.1. Macroscopic Evaluation

Free radical solution polymerization technique was adopted to formulate HPMC-co-AA hydrogel nanoparticles. Prepared composites appeared white colored and sticky with apparent uniform colloidal output.  Figure 2(c) typifies fabricated nanogels with the said characteristics.

### 3.2. Particle Size and Zeta Potential

Fabricated HPMC-based nanocomposites were analyzed for particle size and zeta potential measurement. Figures 2(a) and 2(b) delineate particle size and charge measurements of HPMC nanogels, respectively. Particle diameter turned out to be 117 nm, and PDI was recorded as 0.306. Small polydispersity index (PDI) value indicated that the developed nanogels were homogeneous [33]. Stability and low coagulation tendency of nanogels by electrostatic repulsiveness is authenticated by low zeta potential value (–32). Previously, HPMC-based nanoparticulate systems were reported to have particles size in the range of 38-78 nm [34] and 200 nm [35].

### 3.3. Scanning Electron Microscopy

Surface articulation of formulated cross-linked nanocomposites was evaluated by SEM. Micrographs of analyzed samples are shown in Figures 2(d) and 2(e) for unloaded and FIN-loaded composites, respectively. SEM images portray irregular amorphous texture profile which solidify the stable nanogel formation. Micrograph of FIN-loaded formulation affirms drug trapping in HPMC nanogels.

### 3.4. FTIR Analysis

Developed HPMC-based unloaded and FIN-loaded nanogels along with pure components were analyzed by FTIR in order to identify various functional groups and colligate any interaction among drug and drug carrier system. FTIR spectra of pure HPMC, AA, MBA, FIN, developed nanogels, and FIN-loaded nanogels are given in Figure 3.

FTIR spectrum of HPMC displayed characteristic –OH stretching vibrations at 3483.82 cm^−1^. Methyl and propyl groups were identified at 2901.30 cm^−1^. The spectra showed 6C cyclic ring peak at 1656.54 cm^−1^. The peak at 1374.31 cm^−1^ is associated to C–O–C symmetric bending of methoxy group, and pyranose ring was recognized by a peak at 1053.18 cm^−1^ [36]. FTIR spectra of AA presented characteristic C=C and C–H peaks at 2661.74 cm^−1^ and 2975.73 cm^−1^, respectively. Intense COO^–^ peaks are pointed at 1410.73 and 1616.51 cm^−1^. The carboxyl dispersion band was recognized at 1710.57 cm^−1^. The peak at 1296.89 cm^−1^ is attributed to C–O stretching vibration [37]. FTIR scan of MBA exhibited stretching N–H vibration at 3301.58 cm^−1^, and stretching frequencies of C=O and N–H groups of acryl amide may be attributed to the peaks in the range of 1538.96–1770.21 cm^−1^ [38]. FTIR spectra of FIN expressed alkyl, ketone, and tertiary butyl groups at 1364.17, 1407.98, and 1383.46 cm^−1^, respectively. Peaks for amides I and II were recognized at 1687.05 cm^−1^ and 1600.54 cm^−1^, respectively [39].

The article "Synthesis and Evaluation of Finasteride-Loaded HPMC-Based Nanogels for Transdermal Delivery: A Versatile Nanoscopic Platform" was retracted in 2024. Reasons: signs of a paper mill; compromised peer review; unreliable results or conclusions.

Patternize output for shifting of specific peaks in FTIR spectrum of HPMC nanogels confirmed the successful development of cross-linking network among constituents. Peaks for pure constructive components, i.e., –OH stretching vibrations at 3483.82 cm^−1^, methyl and propyl groups at 2901.30 cm^−1^, C–O–C at 1374.31 cm^−1^, carbonyl dispersion at 1710.57 cm^−1^, intense COO^–^ stretch band at 1616.51 cm^−1^, C–H at 2975.73 cm^−1^, C=C at 2661.74 cm^−1^, C–O at 1296.89 cm^−1^, N–H stretching at 3301.58 cm^−1^, and C=O acryl amide frequency at 1655.78 cm^−1^, were shifted to 3305.61, 2969.74, 1384.49, 1716.46, 1625.26, 2835.56, 2360.88, 3064.10, and 1686.64 cm^−1^, respectively. This overlapping and shifting of characteristic spectral peaks verified formation of successful cross-linked network. Previous data shows the absence and shifting of components specific peaks in HPMC-based formulation [40]. Presence of drug specific peaks was verified by the FTIR scan of FIN-loaded nanogels. The peaks for amide I, amide II, alkyl, ketone, and butyl groups were indicated at 1657.71, 1598.78, 1364.11, 1412.59, and 1385.18 cm^−1^, respectively. Slight shift in peaks of FIN confirmed its successful entanglement in developed nanogels [39].

### 3.5. Thermal Analysis

DSC and TGA of pure constituents and developed nanogels were conducted to inquire the thermal stability and to collect data in context of possible interaction among constituents of the formulation as shown in Figure 4. In DSC scan of pure polymer, endothermic peak starting at 225°C indicates relaxation of polymeric chain. The phase transition temperature is pointed at 320°C. Combustion of polymer is revealed by slight exothermic peak in the range of 325-400°C [41]. DSC spectra of FIN exhibit sharp and prominent peak at 242°C indicating drug melting point and expressing anhydrous crystalline nature of FIN [42]. DSC scan of nanogels showed stable and packed product formation. It was affirmed by the output variation of heat scan of formulated nanogels when compared to pure constituents. Broad endotherm ranging between 30 and 140°C points out the initiation of looseness in polymeric network strands. A broad range of thermal scans also hint the amorphous nature of sample. Evaporation of volatile parts is indicated by an exothermic peak at 275°C. Another exothermic peak at 335°C expresses the glass transition temperature (*T*_*g*_). The endothermic dip at 380°C indicates the nanogel degradation.

The article "Synthesis and Evaluation of Finasteride-Loaded HPMC-Based Nanogels for Transdermal Delivery: A Versatile Nanoscopic Platform" was retracted in 2024. Reasons: signs of a paper mill; compromised peer review; unreliable results or conclusions.

Shifting of thermal peaks and melting temperature (*T*_*m*_) explains a ponderable point that by formation of nanocomposites, the crystalline entities are either converted to or masked by amorphous portion, thus confirming a stable cross-linked system formation. Variation in characteristic endotherm of FIN evidences the successful encapsulation of active ingredient in nanogel network. Previous studies in literature also assert shifting and loss of characteristic endothermic peaks in HPMC-based DDS [43, 44].

TGA scan of HPMC in Figure 4 demonstrates the loss in weight of polymer in three stages. 10% weight loss was noticed in the first stage in the temperature range of 30-210°C. Significance decomposition (80%) of remaining polymer occurred in the range of 211-315°C. The remaining polymeric leftover was degraded in the third stage in the broad temperature range of 325-450°C indicating amorphousness of substance [44, 45]. TGA thermogram of FIN exhibited immediate degradation in the range of 250-300°C which also reveals the crystalline nature of drug [42, 46]. TGA spectra of formulated nanocarrier system portrayed relatively prolonged resistance to thermal decomposition in comparison to those of pure constructive entities. Initial 10% loss of weight occurred from 20 to 225°C indicating the chain relaxation of network. Degradation of major portion of carbon precursor (70%) of nanocomposites is attributed to the detained weight loss in temperature range of 310-390°C. Remaining degradation occurred in temperature higher than 400°C conferring to shrinkage and loss of cross-linking network.

Highly stable nanogel formation is signified by TGA details of composites because of cross-linking network establishment among components when compared to TGA of pure constituents of the formulation. The encapsulation of drug in prepared nanocomposites is also justified by shift in TGA scan when compared to pure FIN. The reason is, when a foreign molecule, i.e., drug moiety, is loaded in the formulated carrier network, its specific thermal characteristics like MP and BP either disappear entirely or make a shift to another temperature range [47]. Enhanced thermal stability of various HPMC-based systems is reported in literature by comparison of thermal scans of constructive entities and developed formulations [48, 49].

The article "Synthesis and Evaluation of Finasteride-Loaded HPMC-Based Nanogels for Transdermal Delivery: A Versatile Nanoscopic Platform" was retracted in 2024. Reasons: signs of a paper mill; compromised peer review; unreliable results or conclusions.

### 3.6. X-Ray Diffraction Studies

X-ray diffraction analysis of fabricated nanocomposites and pure components was performed to uncover the information regarding identification of crystalline or amorphous forms of samples. Scans are presented in Figure 4. XRD scan of pure HPMC exhibits characteristic broad peak at 2*θ* scale value 20 [50, 51]. XRD spectra of pure FIN confirmed crystalline nature of FIN by demonstration of notable distinct and sharp peaks at 2*θ* values of 6, 11, 13, 17, and 19 [12, 52].

Investigation of XRD spectra of developed composites unveils conversion of crystalline form to amorphous entities imprinting the formation of cross-linking network. Successful encapsulation of drug in porous nanogel network was corroborated by absence of specific FIN crystalline spectral peaks. Dissolution of dosage form is also influenced by amorphous or crystalline output. Among the said forms, the former shall produce a relatively fast dissolution rate due to possession of higher internal energy and accreting upsurge molecular motion [53]. Previously, stability of HPMC-based formulations has been reported to be evaluated by XRD [54].

### 3.7. Yield, Sol-Gel, and Porosity Analysis

Percent yield of all prepared nanocomposites came out to be higher than 70%, which insinuates the practical efficiency and impact of method to formulate nanogels. Output of diversity in polymeric, monomeric, and cross-linker content on %yield, sol-gel, and porosity is given in Figure 5. Increase in polymeric concentration in feed ratio of nanogels resulted in higher %yield and gel output. This is attributed to the effect of increased constructive density of developed nanocomposites [55]. Higher %yield and gel were calculated with increase in content of AA. Uplifting the content of constructive entities leads to higher outcome of the said parameters. This could be linked to induction of more free active sites for reaction by availability of activated free radicals for the monomer portion [56]. In the same manner, variation in MBA concentration also influenced the %yield and gel outcome. It is evident from the results that the presence of more cross-linking nodes elevated the cross-link density of fabricated composites that ended up in increased yield and gel content [57].

Results of analysis of porosity of nanocomposites are mentioned in Figure 5 which illustrates that increased HPMC and AA content increased porosity of composites. This is because HPMC and AA grant higher swellability and formation of porous network owing to their hydrophilic nature [58, 59]. In contrast, variation in MBA concentration on %porosity of fabricated nanocomposites unveiled that more stiff and compact cross-linking network was established because of relatively higher net cross-linking density [60].

The article "Synthesis and Evaluation of Finasteride-Loaded HPMC-Based Nanogels for Transdermal Delivery: A Versatile Nanoscopic Platform" was retracted in 2024. Reasons: signs of a paper mill; compromised peer review; unreliable results or conclusions.

### 3.8. In Vitro Swelling Studies

The impact of variation in concentration of HPMC, AA, and MBA on *in vitro* swelling at pH 5.5 and 7.4 was appraised to simulate the ambiance of skin and blood, respectively. Feed ratio of constituents, cross-linking establishment, and porosity response can mark an influence on *in vitro* swelling phenomenon of designed DDS. The results of swelling response is shown in Figure 5. Measurement of swelling index was comparable at both pH with a higher output of said parameter at pH 7.4. Swelling response of network of nanogels is regulated by the smother and presence of electrically charged entities. Various functional groups are responsible for higher swelling index at alkaline pH (7.4). This is because hydroxyl and carboxylic groups dissociate into ionized form at alkaline pH leading to higher electrostatic repulsion, thus creating more spacious network and ultimately resulting in higher swelling [61]. The effect of variation in HPMC concentration on swelling index narrates that increasing the polymeric content increases the swelling index. This is because HPMC possesses great affinity for aqueous media and its formulations can absorb large amount of water in its porous network [58]. The swelling capacity of HPMC-based formulations is directly proportional to its concentration used [62]. An increase in swelling response was observed when AA was increased. This could be comported to relatively higher content of ionized carboxylic groups, subsequently, higher electrostatic repulsion and increased swelling index [63]. The impact of concentration of cross-linking moiety (MBA) on swelling of developed nanogels was evaluated, which showed decreased swelling response with increase in MBA. This could be linked to lower segmental mobility, stiffness, and increased cross-link density of nanogels [64].

### 3.9. Drug Entrapment Efficiency

Synthesized nanocomposites were evaluated for the capability to encapsulate the drug and effect of varying amount of components was checked; the results are mentioned in Figure 6. The polymers with high molecular weight easily encapsulate low molecular weight drugs [65]. Various mechanisms are reported for drug encapsulation by nanogels but swelling based drug loading standout among these [66]. The higher the swelling ability and porosity of developed composites, the more drug from solution is captured [67]. The results reveal that increasing HPMC content ended with relatively higher FIN encapsulation efficacy in nanogels. It is due to the fact that as porosity and swelling increased, drug encapsulation efficiency of nanogels also increased [68]. Likewise, increasing trend of drug entrapment was observed in case of AA. This output is linked to impact of charged carboxylate ions, higher porosity, and increased swelling capability [69]. Moreover, with an increase amount of MBA, relatively lesser drug was captured in the system because of the formation of relatively compact and denser nanocomposites [70].

The article "Synthesis and Evaluation of Finasteride-Loaded HPMC-Based Nanogels for Transdermal Delivery: A Versatile Nanoscopic Platform" was retracted in 2024. Reasons: signs of a paper mill; compromised peer review; unreliable results or conclusions.

### 3.10. In Vitro Drug Release Studies

*In vitro* drug release from synthesized nanocomposites was evaluated, and the results were quantified at pH 5.5 and 7.4 as shown in Figures 6(b) and 6(c), respectively. Variable output of FIN release from nanocomposites was measured against varying content of synthesizing constituents of nanogels as mentioned in Figure 6(a). Swelling, erosion, and diffusion through nanogels play their role in release of active moiety from nanogels. At higher pH, all of the formulations came out with relatively increased drug release outcome correlating to swelling index of nanogels [71].

It is evident from results that *in vitro* FIN release was directly proportional to HPMC content in the nanogel network. This could be linked to the formation of loose networking mesh as a function of water affinitive portion of HPMC [72]. Similarly, effect of increasing AA content on FIN release expressed relatively higher swelling index because of charged carboxylate ions ultimately leads to increased cumulative FIN release profile [73]. On the other hand, FIN release from nanogels was decreased as MBA content increased in the formulation. This output can be attributed to relatively higher cross-link density in developed network which in turn resulted in the production of a closer network mesh that resisted FIN escape from nanogels [64].

### 3.11. Ex Vivo Skin Permeation Studies

Skin permeation evaluation of all developed nanogel formulations was carried by using Franz diffusion cell. Effect of variation in content of HPMC, AA, and MBA was evaluated which showed promising outcome for %FIN permeation, apparent permeability, and flux (Figure 7). HPMC is an important amphiphilic carrier substance that plays an important part in the penetration of moieties through skin. Amphiphilic substance utilize intercellular channels for infiltration through biological membranes [74]. Carbopol-based composites are reported to have accelerated rate of solute diffusion across biological barriers [75]. The results for effect of variation of HPMC on skin permeation revealed increased permeation pattern with increasing polymeric content. This is because of looseness in mesh of nanogels and amphiphilic nature of polymer [76]. Previously developed HPMC-based drug carrier system has been reported to have increased diffusion across skin with increasing diffusible portion in donor part [77]. Dissociation and repulsion of carboxylic groups of AA at alkaline pH result in the formation of destrangled mesh of network of composites which enhanced permeation of FIN from formulation. Correlation between swelling and penetration of active agent from synthesized formulation is reported in literature by various researchers [78, 79]. Unlike HPMC and AA, the output for FIN penetration across skin was decreased as MBA content of formulation increased. Obvious reason for this response is increased cross-linking density of nanogels [80].

The article "Synthesis and Evaluation of Finasteride-Loaded HPMC-Based Nanogels for Transdermal Delivery: A Versatile Nanoscopic Platform" was retracted in 2024. Reasons: signs of a paper mill; compromised peer review; unreliable results or conclusions.

### 3.12. Stability Studies of Carbopol Gel (CG)

Rheological parameters of fresh, 1, 2, and 3 months stored CG were assessed at diverse temperature range, i.e., 8°C, 25°C, 32°C, and 45°C. Measured apparent viscosity, flow index, and thixotropy values are listed in Table 2.  Figure 8 also represents rheograms of CG. The results of analysis interpret decreasing pattern in rheological findings with time, but that decrease was apparently very slight and nonsignificant. All the findings authenticate potential stability of developed CG.

It is evident from the results that CG resisted alteration in viscosity considerably as a function of temperature, thus possessing good thermal stability. The cross-linked junctions fend abjection of polymeric strands with increase in temperature, thus justifying the stability of cross-linking web network [81]. This decrease in viscosity is also supported by the previous research [82]. Flow index measurement were recorded below 1, which indicates the pseudoplasticity feature of developed CG [83]. Rheograms of CG displayed both patterns (ascending and descending) in flow curves. It can be linked to establishment of hysteresis which is also manifested as “thixotropic loop” [84]. Thixotropy is believed to be one of the desirable characteristics for skin-based DDS. This aids efficient applicability, spreading, and penetrating of the entities dispersed in formulation [85].

### 3.13. Skin Irritation Studies

Optimized HPMC-based nanogels were applied on the skin of shaved albino rabbits in order to evaluate the safety profile. The results of skin irritation analysis are given in Table 3. Satisfying results were observed as no indications of skin irritation were noticed through the course. This can be attributed to biocompatibility of cellulose-based composites [86].

### 3.14. Toxicity Studies

#### 3.14.1. Clinical Manifestation

Various parameters, i.e., body weight, water and food intake, signs of illness, hyperactivity, convulsions, and pain response, were noticed during toxicity evaluation of developed nanogels (NHP-6). The results of the abovementioned clinical parameters are given in Table 4 which demonstrated no significant change in the said outcomes with no mortality in both groups under observation. Overall results substantiate the biocompatibility of applied nanogels which could be linked to nontoxic and biocompatible features of HPMC [87, 88].

The article "Synthesis and Evaluation of Finasteride-Loaded HPMC-Based Nanogels for Transdermal Delivery: A Versatile Nanoscopic Platform" was retracted in 2024. Reasons: signs of a paper mill; compromised peer review; unreliable results or conclusions.

#### 3.14.2. Biochemical Investigation

Safety profile of subjects through toxicity studies can be analyzed by collecting vital data regarding blood and blood-based products. Vital information in the context of pathophysiological status of experimental animals can be gathered through haemopoietic markers [89]. In the present study, blood samples from experimental animals were collected and analyzed in view of toxicity assessment of developed nanogels. Table 3 enlists the results for various biochemical parameters which shows that both groups, i.e., control and nanogels treated, manifested no significant differences between biochemical output values, thus asserting biocompatibility of nanogels [90].

#### 3.14.3. Weight Variation and Histopathology

Keeping in view the toxicological studies, autopsy of rabbits of both groups, i.e., control and nanogels treated, was performed to forecast the effect of dabbed formulation on various organs. All experimental work was performed abiding by guidelines of institute's Pharmacy Research Ethics Committee (PREC). Information about the toxic effects of applied formulation can be collected through output of weight variation and histopathological examination [91]. The results of weight measurement of vital organs of rabbits are enlisted in Table 3 which showed no significant weight variation among the animals in groups under examination. The results of histology of vital body organs, i.e., skin, heart, liver, kidney, and lungs are presented in Figure 7(g). The results articulate normal tissue structure with no sign of pathology which hints the biocompatibility of applied nanogels [92].

## 4. Conclusion

On the basis of the current study, it can be concluded that HPMC-based nanogels were prepared for efficient transdermal drug delivery. Characterization (FTIR, SEM, TGA, DSC, and XRD) confirmed formation of stable composites. In vitro and ex vivo analysis confirmed formation of a stable, effective, and biocompatible drug delivery system. Such transdermal nanogel drug transport structure can be designed to overcome the limitations related to long time oral therapy as well as alternate to invasive drug delivery. Moreover, to avoid the first pass metabolism and promote better outcomes with improved patient compliance. However, in the future, there exists a need to perform *in vivo* studies on human volunteers.

The article "Synthesis and Evaluation of Finasteride-Loaded HPMC-Based Nanogels for Transdermal Delivery: A Versatile Nanoscopic Platform" was retracted in 2024. Reasons: signs of a paper mill; compromised peer review; unreliable results or conclusions.

## Figures and Tables

**Figure 1:** Proposed cross-linked structure of HPMC nanogels.

**Figure 2:** (a) Particle size distribution. (b) Zeta potential. (c) Physical state. (d) SEM micrograph of unloaded. (e) FIN-loaded HPMC-co-AA nanogels.

**Figure 3:** FTIR spectrum of HPMC, AA, MBA, FIN, unloaded, and FIN-loaded HPMC-co-AA nanogels.

**Figure 4:** The spectra of TGA, DSC, and XRD of polymer HPMC, pure drug FIN, and developed composites.

**Figure 5:** Impact of polymer HPMC, monomer AA, and cross-linker MBA variance on percent outcome of gel, yield, porosity, and swelling index.

**Figure 6:** (a) Impact of various components on percent drug entrapment efficiency (%DEE) and percent drug release. (b) Percent drug release of developed nanogels and reference product at pH 5.5. (c) Percent drug release of developed nanogels and reference product at pH 7.4.

**Figure 7:** Effect of (a) HPMC, (b) AA, (c) MBA on % drug permeation, (d) %drug deposited, (e) apparent permeability, (f) flux, and (g) histological examination of various organs of rabbits.

**Figure 8:** Rheograms of carbopol gel (CG) kept at different storage conditions: (a) freshly prepared, (b) after one month, (c) after two months, and (d) after three months.

**(a):** 

Sr. no	Formulation code	HPMC (g/100 g)	Acrylic acid (g/100 g)	APS/SHS (g/100 g)	MBA (g/100 g)
SET-I^∗^					
1	NHP-1	0.8	8	0.8/0.8	8
2	NHP-2	1.6	8	0.8/0.8	8
3	NHP-3	2.4	8	0.8/0.8	8

SET-II^∗∗^					
4	NHP-4	2.4	8	0.8/0.8	8
5	NHP-5	2.4	12	0.8/0.8	8
6	NHP-6	2.4	16	0.8/0.8	8

SET-III^∗∗∗^					
7	NHP-7	2.4	8	0.8/0.8	8
8	NHP-8	2.4	8	0.8/0.8	10
9	NHP-9	2.4	8	0.8/0.8	12

**(b):** 

Studied variables	Variables level (g)		
	Low	Medium	High
C-1^∗^	0.8	1.6	2.4
C-2^∗∗^	8	12	16
C-3^∗∗∗^	8	10	12

Abbreviations: C-1^∗^: HPMC conc.; C-2^∗∗^: AA conc.; C-3^∗∗∗^: MBA conc.

**Table 2:** Apparent viscosity, flow index, and thixotropy of CG.

Parameter	Time	Temp			
Apparent viscosity (dynes/cm^2^)		8°C	25°C	32°C	45°C
	Fresh		291.59		
	(1) Month	287.15	278.37	281.88	280.9
	(2) Month	285.74	282.07	277.48	272.72
	(3) Month	282.94	281.12	275.29	268.12

Flow index	Fresh		0.63		
	(1) Month	0.62	0.62	0.61	0.61
	(2) Month	0.62	0.6	0.61	0.6
	(3) Month	0.63	0.59	0.59	0.58

Thixotropy (dynes/cm^2^.S)	Fresh		7508		
	(1) Month	7480	7331	7325	7283
	(2) Month	7421	7324	7222	7113
	(3) Month	7352	7283	7170	6970

**(a):** 

Irritation test results on rabbits					
Formulation applied		Time of observation			
		24 h	48 h	72 h	240 h
Control	1	—	—	—	—
	2	—	—	—	—
	3	—	—	—	—

HPMC nanogels	1	—	—	—	—
	2	—	—	—	—
	3	—	—	—	—

Irritation scale					
Sign	—	+	++	+++	++++
Outcome	None	Very slight	Well defined	Moderate	Eschar formation

**(b):** 

Liver, kidney, and lipid profile		
Parameter	Control	Nanogels
ALT (SGPT) (U/l)	117 ± 8.26	129 ± 12.17
AST (SGOT) (U/l)	71 ± 4.91	78 ± 4.81
Serum urea (mg/dl)	14.3 ± 0.94	14.8 ± 0.77
Serum creatinine (mg/dl)	0.8 ± 0.11	0.7 ± 0.12
Serum uric acid (mg/dl)	2.9 ± 0.24	3 ± 0.21
Total cholesterol (mg/dl)	58 ± 3.16	63 ± 3.19
Triglycerides (mg/dl)	45 ± 2.49	49 ± 3.08

**(c):** 

Effect of nanogel administration on organ weights (g) of rabbits (*n* = 3)					
Groups	Heart	Liver	Lung	Kidney	Spleen
Control	4.63 ± 0.11	79.42 ± 0.17	9.33 ± 0.26	12.63 ± 0.24	1.03 ± 0.14
Nanogels	4.79 ± 0.11	81.94 ± 0.14	9.53 ± 0.17	13.11 ± 0.23	1.15 ± 0.21

**(d):** 

Haematological analysis		
Parameter	Control	Nanogels treated
Hb (g/dl)	14.3 ± 0.87	14.4 ± 0.89
pH	7.31 ± 0.04	7.24 ± 0.05
RBCs (×10^6^/mm^3^)	6.41 ± 42436	6.44 ± 39974
TLC (×10^3^/mm^3^)	9.2 ± 199.64	9.3 ± 232.17
Eosinophil (%)	2.1 ± 0.19	2.2 ± 0.19
Neutrophils (%)	49.2 ± 2.19	51.6 ± 1.86
Monocytes (%)	2.7 ± 0.22	2.9 ± 0.29
Lymphocytes (%)	58.3 ± 2.24	63.5 ± 2.58
PLT (×10^3^/mm^3^)	339 ± 5.14	352 ± 5.81
MCV (fl)	64.4 ± 3.28	64.9 ± 2.53
MCH (pg/cell)	19.2 ± 1.11	19.4 ± 1.22
MCHC (g/dl)	30.0 ± 1.73	30.7 ± 1.51

Values expressed as mean ± SD, *n* = 3.

The article "Synthesis and Evaluation of Finasteride-Loaded HPMC-Based Nanogels for Transdermal Delivery: A Versatile Nanoscopic Platform" was retracted in 2024. Reasons: signs of a paper mill; compromised peer review; unreliable results or conclusions.

**Table 4:** Clinical observations of toxicity studies.

Parameter observed	Time for observation	Group I (control)			Group III (treated with HPMC nanogels) 500 mg/kg of body weight		
Body weight (kg)	Pretreatment	2.17 ± 0.08			2.19 ± 0.03		
	24 h	2.19 ± 0.12			2.20 ± 0.05		
	48 h	2.18 ± 0.11			2.21 ± 0.03		
	72 h	2.19 ± 0.13			2.22 ± 0.06		
	240 h	2.19 ± 0.17			2.24 ± 0.02		

Food intake (g/day)	Pretreatment	63 ± 10.71			67 ± 7.62		
	24 h	62 ± 13.87			64 ± 9.24		
	48 h	61 ± 8.93			60 ± 5.75		
	72 h	63 ± 11.24			70 ± 7.53		
	240 h	58 ± 9.54			63 ± 9.48		

Water intake (ml/day)	Pretreatment	162 ± 11.72			179 ± 20.74		
	24 h	175 ± 6.89			178 ± 18.45		
	48 h	157 ± 45.34			176 ± 19.67		
	72 h	163 ± 12.82			169 ± 15.09		
	240 h	172 ± 23.09			187 ± 20.42		

		R1	R2	R3	R1	R2	R3
Signs of illness	Pretreatment	0	0	0	0	0	0
	24 h	0	0	0	0	0	0
	48 h	0	0	0	0	0	1
	72 h	0	0	0	0	1	0
	240 h	0	0	0	0	0	0

Convulsion	Pretreatment	0	0	0	0	0	0
	24 h	0	0	0	0	0	0
	48 h	0	0	0	0	0	0
	72 h	0	0	0	0	0	0
	240 h	0	0	0	0	0	0

Hyperactivity	Pretreatment	0	0	0	0	0	0
	24 h	0	0	0	0	0	1
	48 h	0	0	2	1	0	0
	72 h	0	0	0	0	1	0
	240 h	0	0	0	0	0	1

Pain response	Pretreatment	1	1	1	1	1	1
	24 h	1	1	1	1	1	1
	48 h	1	0	1	0	1	1
	72 h	1	1	1	1	1	0
	240 h	1	1	1	1	1	1

Scale	Sign			0	1	2	3
	Outcome			Absent	Mild	Moderate	Intense

## Data Availability

The data used to support the findings of this study are included within the article.

The article "Synthesis and Evaluation of Finasteride-Loaded HPMC-Based Nanogels for Transdermal Delivery: A Versatile Nanoscopic Platform" was retracted in 2024. Reasons: signs of a paper mill; compromised peer review; unreliable results or conclusions.

## Supplementary Materials

Supplementary Materials Graphical abstract exhibits the preparation technique, characterization, and toxicity evaluation of the developed nanogels.
